The article "Establishment of Normal Range for Thromboelastography in Healthy Middle-Aged and Elderly People of Weihai in China" was published in 2021. Journal: J Healthc Eng.

# Establishment of Normal Range for Thromboelastography in Healthy Middle-Aged and Elderly People of Weihai in China

**DOI:** 10.1155/2021/7119779

**Published:** 2021-11-28

**Authors:** Lina Ni, Peng Xue, Changjuan An, Xia Yu, Jiangli Qu, Yingjie Yao, Yingbo Li

**Affiliations:** Department of Blood Transfusion, Weihai Central Hospital, Weihai 264200, Shandong Province, China

## Abstract

TEG can monitor the dynamic changes of blood clot formation and lysis by activating the coagulation system of a small sample of whole blood in vitro. The parameters can reflect the level of coagulation factors, the function of fibrinogen and platelet, and the presence or absence of hyperfibrinolysis. At present, the normal reference range of the parameters of TEG is mainly based on the reference values established by the Western population. Due to the differences in the distribution of ethnic groups, many countries have established their reference ranges for healthy populations. In China, some scholars have tried to establish the corresponding TEG reference range according to the characteristics of the population in different regions. This study tried to establish the reference range for thromboelastography in healthy middle-aged and elderly people of Weihai in China and compare it with the reference range provided by the manufacturer. The fasting venous blood of 454 healthy middle-aged and elderly people was collected, including 239 males and 215 females. The thromboelastography TEG-5000 was used to measure the reaction time (R), coagulation formation time (K), coagulation angle (Angle), and maximum amplitude (MA). The reference range of TEG parameters of middle-aged and elderly healthy males was R: 4.38–8.27 min, K: 1.44–2.82 min, Angle: 48.53–72.17 deg, and MA: 51.95–72.02 mm; respectively, in the females, the normal value was R: 3.43–7.40 min, K: 1.07–2.53 min, Angle: 48.22–77.22 deg, and MA: 53.10–74.58 mm; The difference of R, K, Angle, and MA between the male group and the female group was statistically significant (*P* < 0.05); In this study, if we use the reference range established by the manufacturer, the R specificity for males was 91.6%, K specificity was 98.7%, Angle specificity was 85.8%, and MA specificity was 93.7%; the range for females was 68.4%, 99.5%, 75.8%, and 87.4%, respectively. There are statistically significant differences between R, K, Angle, and MA in middle-aged and elderly healthy women and men. It is necessary to establish a TEG reference range for healthy females and males.

## 1. Introduction

Thromboelastography (TEG) was invented by the German Harter in 1948. TEG can monitor the dynamic changes of blood clot formation and lysis by activating the coagulation system of a small sample of whole blood in vitro. The parameters can reflect the level of coagulation factors, the function of fibrinogen and platelet, and the presence or absence of hyperfibrinolysis [1]. TEG is of great significance in determining the cause of bleeding in patients, assessing perioperative risk, and monitoring the effect of anticoagulant drugs. The traditional coagulation tests such as PT, APTT, Fg, and TT only detect part of the blood coagulation components in the plasma and cannot evaluate the function of whole blood. So, it is not possible to comprehensively and accurately determine the abnormality of the body's blood coagulation system. Wang et al. believe that TEG is superior to traditional coagulation tests in assessing the hypercoagulable state and bleeding risk of patients with prostate cancer [2]. Terada et al. compared the methods of assessing the risk of bleeding after cardiac surgery and the effect of platelet transfusion; the results showed that TEG was better. TEG was originally mainly used to monitor coagulation changes in liver transplantation [3]. After decades of development, TEG has been widely used in various fields of cardiac surgery [4], postpartum hemorrhage, hemophilia, and brain trauma surgery [5, 6]. At present, the normal reference range of the parameters of TEG is mainly based on the reference values established by the Western population. Due to the differences in the distribution of ethnic groups, many countries have established their own reference ranges for healthy populations [1, 7]. In China, some scholars have tried to establish the corresponding TEG reference range according to the characteristics of the population in different regions [8, 9]. This study tried to establish the reference range for thromboelastography in healthy middle-aged and elderly people of Weihai in China and compared it with the reference range provided by the manufacturer.

The article "Establishment of Normal Range for Thromboelastography in Healthy Middle-Aged and Elderly People of Weihai in China" was published in 2021. Journal: J Healthc Eng.

## 2. Materials and Methods

### 2.1. Inclusion Criteria of Healthy Subjects

The study was conducted at the Central Hospital of Weihai with middle-aged and elderly volunteers (age ≥45 years), residents of Weihai China. The results of liver function, renal function, fasting blood glucose, and serum lipid and routine blood tests were within the normal reference ranges of the lab. The pregnant women, menstrual women, patients with a history of bleeding or thrombosis, those taking anticoagulant drugs (warfarin, rivaroxaban, argatroban, etc.) or antiplatelet drugs (aspirin, bolivive, etc.), and those who have suffered from other diseases (including colds) in the past six months were excluded. After recruitment, healthy subjects were divided into two groups according to their gender. The study was approved by the Ethics Committee of Weihai Central Hospital.

### 2.2. Collection of Samples and Basic Information

Early morning whole blood samples were collected smoothly in sodium citrate- and EDTA-K_2_-anticoagulated vaccutainers, respectively. The vaccutainers were gently reversed in time to make the blood and anticoagulant thoroughly mix, and samples were centrifuged. The samples for TEG were incubated at 37°C for 15 minutes. According to the inclusion criteria, exclusion criteria, and relevant test results, 32 volunteers were excluded. Eventually, 454 middle-aged and elderly volunteers were included in this study, with 239 males and 215 females.

### 2.3. TEG Analysis

The sodium citrate-anticoagulated whole blood was incubated at 37°C for 15 minutes in accordance with the operating procedures. At the same time, kaolin (Haemoscope Corp, USA) was removed from the storage refrigerator and restored to room temperature. Following specimen and reagent preparation, we added a 1.0 ml sample to the kaolin cup along the wall and gently mixed it according to the operating procedures. We then install the ordinary test cup on the machine and added 20 *μ*l 0.2 M of calcium chloride, drew 340 microliters of kaolin-activated whole blood into the cup, pushed the cup up, kept the control lever in the test position, and started running the specimen until the MA value was determined [10]. A TEG-5000 analyzer (Haemoscope Corp, USA) was used to get the main parameters including R, K, Angle, and MA. The computer-controlled TEG-5000 analyzer automatically analyzed the dynamics of coagulation and fibrinolysis in the form of a graph, and the result of coagulation status is obtained by a comprehensive analysis of the measured parameters.

### 2.4. Statistical Analysis

Data analysis was performed using SPSS 19.0 statistical software package (SPSS Inc., Chicago, IL). The parameters were compared using the *t*-test and Mann–Whitney *U* test as appropriate. Normality of the data was tested with the Kolmogorov–Smirnov test, while correlations were determined by Spearman's rank correlation coefficients. All tests were two-sided, and the difference was statistically significant when the *P* value was less than 0.05.

## 3. Results

### 3.1. General Information of Healthy Volunteers

We grouped 454 volunteers who met the entry criteria into two groups according to gender. The basic information of the two groups of volunteers was compiled, as shown in Table 1.

### 3.2. Internal Quality Control of TEG

We used 3 TEG-5000 thromboelastography analyzers (Haemoscope Corp, USA) for a total of 6 detection channels. Level 1 and Level 2 quality control materials were determined on 6 channels each day as shown in Tables 2 and 3.

The article "Establishment of Normal Range for Thromboelastography in Healthy Middle-Aged and Elderly People of Weihai in China" was published in 2021. Journal: J Healthc Eng.

### 3.3. Assessment of TEG Results in Two Groups

In this study, healthy middle-aged and old people were grouped by gender. The results showed that R, K, Angle, and MA of TEG-5000 had statistically significant differences between males and females, as shown in Table 4. We analyzed the data and established the reference range of the subjects included in this study for main parameters of TEG, as shown in Table 5.

### 3.4. Assessment of the Reference Range Provided by Manufacturers

To assess whether the reference range provided by manufacturers is appropriate to the subjects included in this study, we analyzed the application value. When the normal range provided by the manufacturer was used, R, K, Angle, and MA values of 239 male healthy volunteers were 8.4%, 1.3%, 14.2%, and 6.3%, respectively, out of the range provided. Among female healthy volunteers, the values exceeded the manufacturer reference by 31%, 0.5%, 24.2%, and 12.6% for R, K, Angle, and MA, respectively, as shown in Table 6.

## 4. Discussion

According to the reference range provided by the manufacturers, the specificity of K value in males and females was 98.7% and 98.7%, respectively, reaching the expected accuracy of 95%, but the specificity of R, Angle, and MA was all below 95%. In the female group, the specificity of R and Angle was 68.4% and 75.8%, respectively. Scarpelini et al. provided similar reports. The false-positive rates of R, K, Angle, and MA they reported were 16.9%, 5.9%, 12.7%, and 12.7% [1]. It is suggested that if the reference range provided by the manufacturer is used, there will be a false-positive rate report of 0.5%–31.6% for each parameter in this study. This may lead to an opposite diagnosis of coagulation abnormalities or incorrect blood transfusion treatment. Therefore, it is necessary to establish an appropriate TEG reference range for healthy people in various regions [11]. This study found that the values of TEG parameters R, K, Angle, and MA are related to gender. Women's R and K values are lower than men's, but their Angle and MA values are higher than men's. This result is consistent with the findings of other scholars [7, 9, 12], suggesting that middle-aged and elderly female have stronger coagulation functions than males.

Qin et al. [13] studied the changes in TEG parameters of newborns (≥37 weeks of pregnancy) and developed reference ranges for newborns: R: 2.8–7.17, K: 0.8–4.5, Angle: 44.91–78.89, and MA: 44.34–74.66 and found that as age increases, Angle and MA increased and *K* values decreased; Mirabella et al. believed that there is no significant difference in TEG parameters between newborns and adults [14]; Motta et al. used TEG to test the coagulation function of early preterm infants and mid-to-late stage neonates. They believed that there was no significant difference between the two. Although the levels of coagulation factors and anticoagulation factors were low in preterm infants, the coagulation function was stable [15]. Antony KM found that the coagulation function of pregnant women was stronger than that of the adult group [16]. Gui et al. found that the blood coagulation in pregnant women was related to blood type. The *R* value of type O pregnant women was longer than that of non-type O pregnant women, suggesting that type O pregnant women had a higher risk of bleeding during delivery [9]. Patients with advanced liver disease have low expression of coagulation factors. De Pietri et al. found that the TEG results of patients with liver cirrhosis are significantly different from those of the normal population, and it is considered necessary to establish a TEG reference range for this type of disease [17].

The article "Establishment of Normal Range for Thromboelastography in Healthy Middle-Aged and Elderly People of Weihai in China" was published in 2021. Journal: J Healthc Eng.

## 5. Conclusion

In the future, we will conduct research on healthy children, pregnant women, elderly, and various diseases in Weihai to establish reference ranges, needed to improve the level of judgment in patients with coagulation abnormalities and offer guidance to clinical blood transfusion. There were not enough volunteers recruited in this study, and the scope of the investigation and research in this area is not comprehensive enough. The domestic TEG internal quality evaluation has not been fully carried out, which may have some impact on the establishment of the TEG reference range. In the future, we will continue to recruit more healthy middle-aged and elderly people in the region and continue to improve the established reference range.

In summary, we established reference ranges for different TEG parameters in Weihai, China. This study has provided more accurate information needed for future scientific research in the field of blood coagulation.

## Figures and Tables

**Table 1:** Clinical information of healthy volunteers.

Parameters	Male (*N* = 239)	Female (*N* = 215)
Age (year)	60.40 ± 8.79	61.40 ± 9.66
ALT (U/L)	17 (21–28)	15 (19–24)
AST (U/L)	19 (21–24)	16 (19–21)
TP (g/L)	70.71 ± 3.30	71.96 ± 4.81
Alb (g/L)	45.57 ± 2.56	45.06 ± 2.36
Urea (mmol/L)	5.20 ± 1.01	4.77 ± 1.022
Crea (*µ*mol/L)	66.00 ± 7.16	56.05 ± 8.34
FBS (mmol/l)	4.94 ± 0.56	5.05 ± 0.56
TC (mmol/L)	4.17 ± 0.56	4.28 ± 0.53
TG (mmol/L)	1.03 ± 0.33	1.09 ± 0.32
RBC (10^12^/L)	4.85 ± 0.38	4.41 ± 0.29
WBC (10^10^/L)	6.67 ± 1.37	6.02 ± 1.23
Hb (g/L)	149.04 ± 10.32	130.84 ± 8.78
PLT (10^9^/L)	209.23 ± 42.96	214.65 ± 41.23

ALT: alanine transferase, AST: aspartate transferase, TP: total protein, Alb: albumin, Crea: creatinine, FBS: fasting blood sugar, TC: total cholesterol, TG: triglycerides, RBC: red blood cell count, WBC: white blood cell count total, Hb: hemoglobin, and PLT: platelet count.

The article "Establishment of Normal Range for Thromboelastography in Healthy Middle-Aged and Elderly People of Weihai in China" was published in 2021. Journal: J Healthc Eng.

**Table 2:** Internal quality control analysis of Level 1 for 30 consecutive days.

	*R* (min)	*K* (min)	Angle (deg)	MA (mm)
Channel 1	1.53 ± 0.08 (5.2%)	0.80 ± 0.06 (7.5%)	83.13 ± 0.75 (0.9%)	52.83 ± 5.06 (9.5%)
Channel 2	1.55 ± 0.14 (9.0%)	0.83 ± 0.05 (6.0%)	81.9 ± 0.71 (0.8%)	54.18 ± 5.32 (9.8%)
Channel 3	1.58 ± 0.12 (7.5%)	0.81 ± 0.05 (6.1%)	82.24 ± 1.30 (1.5%)	50.16 ± 5.01 (9.9%)
Channel 4	1.60 ± 0.09 (5.6%)	0.80 ± 0.06 (7.5%)	82.02 ± 2.65 (3.2%)	51.38 ± 5.10 (9.9%)
Channel 5	1.57 ± 0.05 (3.1%)	0.80 ± 0.03 (3.7%)	82.83 ± 2.09 (3.2%)	52.08 ± 5.04 (9.6%)
Channel 6	1.59 ± 0.06 (3.7%)	0.80 ± 0.04 (5.0%)	82.18 ± 1.48 (1.8%)	52.88 ± 5.20 (9.8%)
Reference range	0–4	0–2	76–88	42–62

The number in brackets is the coefficient of variation.

**Table 3:** Internal quality control analysis of Level 2 for 30 consecutive days.

	*R* (min)	*K* (min)	Angle (deg)	MA (mm)
Channel 1	1.32 ± 0.04 (3.0%)	0.82 ± 0.06 (7.3%)	75.04 ± 0.72 (0.8%)	32.61 ± 0.95 (2.9%)
Channel 2	1.30 ± 0.08 (6.1%)	0.81 ± 0.04 (4.9%)	74.88 ± 0.85 (1.0%)	32.28 ± 1.19 (3.6%)
Channel 3	1.32 ± 0.07 (5.3%)	0.80 ± 0.03 (3.7%)	75.34 ± 1.42 (1.7%)	33.04 ± 1.09 (3.2%)
Channel 4	1.50 ± 0.07 (4.6%)	0.81 ± 0.04 (4.9%)	74.77 ± 1.09 (1.3%)	32.34 ± 1.75 (5.4%)
Channel 5	1.37 ± 0.09 (6.5%)	0.80 ± 0.02 (2.5%)	75.65 ± 0.47 (0.5%)	33.27 ± 0.49 (1.4%)
Channel 6	1.35 ± 0.05 (3.7%)	0.81 ± 0.04 (4.9%)	75.00 ± 0.66 (0.8%)	32.60 ± 1.84 (5.6%)
Reference range	1–3	0–5	57–80	25–40

The number in brackets is the coefficient of variation.

**Table 4:** Comparison of main parameters of TEG-5000 in middle-aged and elderly males and females (*x* ± *s*).

Parameters	Male (*N* = 239)	Female (*N* = 215)
*R* (min)^∗^	6.33 ± 0.99	5.41 ± 1.01
*K* (min)^∗^	2.13 ± 0.35	1.80 ± 0.37
Angle (deg)^∗^	60.35 ± 6.03	62.72 ± 7.40
MA (mm)^∗^	61.99 ± 5.12	63.84 ± 5.48

^∗^There is a significant difference between the two groups (*P* < 0.05).

**Table 5:** Reference range of TEG-5000 for middle-aged and old males and females in this study (*x* ± 1.96 s).

Parameters	Male (*N* = 239)	Female (*N* = 215)
*R* (min)	4.38–8.27	3.43–7.40
*K* (min)	1.44–2.82	1.07–2.53
Angle (deg)	48.53–72.17	48.22–77.22
MA (mm)	51.95–72.02	53.10–74.58

**Table 6:** Assessment of the reference range provided by manufacturers.

Reference range provided by manufacturers								
	*R* (5–10) min		*K* (1–3) min		Angle (53–72) deg		MA (50–70) mm	

Result	+	−	+	−	+	−	+	−
Male	20 (8.4%)	219 (91.6%)	3 (1.3%)	236 (98.7%)	34 (14.2%)	204 (85.8%)	15 (6.3%)	224 (93.7%)
Female	68 (31.6%)	147 (68.4%)	1 (0.5%)	214 (99.5%)	52 (24.2%)	163 (75.8%)	27 (12.6%)	188 (87.4%)

Note: +, out of the reference range provided by manufacturers; −, within the reference range provided by manufacturers. Numbers in brackets indicate the proportion.

The article "Establishment of Normal Range for Thromboelastography in Healthy Middle-Aged and Elderly People of Weihai in China" was published in 2021. Journal: J Healthc Eng.

## Data Availability

The datasets used and/or analyzed during the current study are available from the corresponding author on reasonable request.

## Abbreviations

TEG: Thromboelastography
R: Reaction time
K: Clot kinetics
Angle: Fibrin production rate
MA: Maximum amplitude
PT: Prothrombin time
APTT: Activated partial thromboplastin time
Fib: Fibrinogen
TT: Thromboplastin time
TP: Total protein
Alb: Albumin
ALT: Alanine transferase
AST: Aspartate transferase
Urea: Urea nitrogen
Crea: Creatinine
TC: Total cholesterol
TG: Triglycerides
FBS: Fasting blood sugar
PLT: Platelet count
RBC: Red blood cell
WBC: White blood cell count total
Hb: Hemoglobin.
